# Lower-Limb-Assisting Robotic Exoskeleton Reduces Energy Consumption in Healthy Young Persons during Stair Climbing

**DOI:** 10.1155/2021/8833461

**Published:** 2021-04-24

**Authors:** Hanseung Woo, Kyoungchul Kong, Dong-wook Rha

**Affiliations:** ^1^Department of Mechanical Engineering, Korea Advanced Institute of Science and Technology (KAIST), Daejeon 34141, Republic of Korea; ^2^Angel Robotics, Seoul 04798, Republic of Korea; ^3^Department and Research Institute of Rehabilitation Medicine, Yonsei University College of Medicine, Seoul 03722, Republic of Korea

## Abstract

Many robotic exoskeletons for lower limb assistance aid walking by reducing energy costs. However, investigations examining stair-climbing assistance have remained limited, generally evaluating reduced activation of related muscles. This study sought to investigate how climbing assistance by a robotic exoskeleton affects energy consumption. Ten healthy young participants wearing a robotic exoskeleton that assists flexion and extension of hip and knee joints walked up nine flights of stairs twice at a self-selected speed with and without stair-climbing assistance. Metabolic cost was assessed by measuring oxygen consumption, heart rate, and the time to climb each flight of stairs. Net oxygen cost (NOC) and total heart beats (THB) were used as measures of metabolic cost, accounting for different climbing speeds. Stair-climbing assistance reduced NOC and THB by 9.3% (*P* < 0.001) and 6.9% (*P* = 0.003), respectively, without affecting climbing speed. Despite lack of individual optimization, assistive joint torque applied to the hip and knee joints reduced metabolic cost and cardiovascular burden of stair climbing in healthy young males. These results may be used to improve methods for stair ascent assistance.

## 1. Introduction

Various robotic exoskeletons for lower limb assistance have been developed to aid walking, the most common method of human locomotion. Investigations of walking mechanics have provided the foundation for the development of such robots. Kinematics of lower limb joints have been used to determine the range of motion and the degree of freedom of robotic joints [1], whereas kinetics have been used to determine the required robot joint power [2]. Together, kinematics and kinetics have provided important insights into the development of appropriate walking assistance methods.

The benefits of walking assistance provided by robotic exoskeletons have been evidenced as reduced energy costs. For instance, ankle exoskeletons utilizing pneumatic muscles to assist ankle plantar flexion have been shown to reduce the metabolic cost of walking [3–5]. However, these exoskeletons were not fully mobile, as they were powered by an external air pressure source, with the energy cost advantage observed only on a treadmill at a constant walking speed.

The metabolic cost benefits of the portable autonomous ankle exoskeleton developed by Mooney et al. [6, 7] were similarly verified in a controlled environment. Recent studies demonstrated that walking assistance by a tethered multijoint soft exosuit significantly reduced metabolic costs [8, 9]. Furthermore, an autonomous version of the soft exosuit reduced the metabolic cost of walking together with a carrying load [10, 11]. In a case study of overground walking assistance with two subjects, the autonomous soft exosuit also reduced the metabolic cost of loaded walking over a 500 m cross-country trail [12].

Although stair climbing is almost as frequent as walking, the biomechanical characteristics of the two types of motion are distinct from each other. Relative to walking, stair climbing, characterized by large joint moment and power, increases joint flexion in the hip, knee, and ankle in the sagittal plane. During stair climbing, power generation in the knee joint is dominant relative to power absorption, and the total positive network of the joints is larger than that during walking [13, 14]. Given that stair climbing requires considerable joint torque, positive power, and positive network, assistance provided by a wearable robot is expected to reduce the energetic cost of ascent by providing assistive torque to the wearer's joints.

Previous reports have proposed climbing assistance methods facilitated by robotic exoskeletons. Despite utilizing different exoskeletons, actuators, sensors, and target users, several studies have verified, using electromyography, the effects of stair-climbing assistance on subjects capable of performing voluntary leg motions [15–17]. Yet, to date, the effects of exoskeleton-mediated climbing assistance on energetic costs have not been considered, with a limited number of studies analyzing the metabolic effects of assistance for other related motions. For instance, assistance provided by a knee exoskeleton during step-up-and-down [18] and squatting [19] exercises has been shown to reduce the heart rate and the metabolic equivalent of task [20], respectively. Presently, we sought to investigate the energy consumption effect of stair-climbing assistance provided by a robotic exoskeleton. Specifically, we tested oxygen consumption and heart rate during a nine-flight stair climb in the absence or presence of assistance from an autonomous (i.e., fully mobile) robotic exoskeleton with rigid frames and braces providing assistive torque to the hip and knee joints.

## 2. Materials and Methods

### 2.1. Participants

Nondisabled male subjects (*N* = 10, age = 28.3 ± 1.7 years, weight = 68.8 ± 5.5 kg, height = 173.8 ± 5.1 cm) participated in this study. None of the subjects have been diagnosed with musculoskeletal or neurologic disorders affecting walking or stair climbing. Ethical approval was granted by the institutional review board and ethics committee (4-2017-0578).

### 2.2. Robotic Exoskeleton

The robotic exoskeleton used in this study (Figure 1) consisted of active hip and knee joints and passive ankle joints. Active joints were powered by electrical motors with a gear ratio of 76 : 1, with assistive torque delivered to the wearer's joints in the sagittal plane. Active joints adopted a series elastic actuation mechanism [21, 22], enabling accurate control of the interaction torque between robot and human joints. Dynamic ankle-foot orthosis was used as the passive ankle joint to support the weight of the exoskeleton and to provide a sufficient degree of freedom in the wearer's ankle joint. Foot pressure under the metatarsal joint and the heel was measured using silicon tubes and air pressure sensors to estimate the ground reaction force [23]. All algorithms required to operate the exoskeleton, such as sensor signal processing and the control algorithm, were implemented using the embedded control board (sbrio 9651, National Instruments, TX, USA) and software (LabVIEW 2015, National Instruments, TX, USA). The embedded control board and battery, enclosed in a backpack, enabled the exoskeleton to be fully mobile. The total weight of the robotic exoskeleton was 13 kg.

### 2.3. Assistance Strategy for a Stair-Climbing Motion

Common robotic joints are actuated by motors and gear reducers to amplify output torque to the desired magnitude. However, such a gear train is associated with large resistive torque. To remove the resistance and allow the wearer to move freely without discomfort, the robotic exoskeleton used a zero-impedance control (ZIC) algorithm [21, 24–26]. As shown in Figure 2, the ZIC application reduced the interaction torque between robotic and human joints such that it lies under 0.87 Nm. Also, it allowed the wearer to move the joint much faster with reduced resistive force.

Following ZIC-mediated removal of resistance, assistive torque can be provided via an assist-as-needed strategy [27, 28], which requires the determination of the timing for the application of the assistive torque. Previous studies [5, 29, 30] have used actuation onset timing, with a predefined assistive force provided at onset timing determined based on the percentages of a gait cycle. Presently, we employed a similar strategy for the stair-climbing assistance.

An investigation by Riener et al. of stair-climbing biomechanics and motor coordination [13] revealed substantial extension torque of the hip and knee joints during the early section of the stance phase. Flexion torques are also observed in both joints during the initial section of the swing phase. The developed assistive joint torque profile for stair climbing emulated the joint torques during the early sections of the stance and swing phases. The assistive torque profile for the hip and knee joints can be simplified and parameterized as

(1) $$\begin{array}{c} \tau_{o}\left(t\right)=\left\{\begin{array}{c} -0.5\left(\tau_{p}\cos\left(\frac{\pi }{t_{p}}\left(t-t_{i}\right)\right)-\tau_{p}\right),\text{if }t\in \left[t_{i},t_{i}+2t_{p}\right],\\ 0,\text{otherwise}, \end{array}\right. \end{array}$$

where *t*_*i*_, *τ*_*p*_, and *t*_*p*_ indicate onset time, peak value of the assistive torque, and time to reach, *τ*_*p*_, respectively. When *τ*_*o*_(*t*) = 0, the desired interaction torque is zero, indicating a zero-impedance mode. Positive and negative values of *τ*_*p*_ indicate extension and flexion torque, respectively. To provide assistive torque during the early section of both phases, *t*_*i*_ can be set as the time when each phase is detected by analyzing the ground reaction forces [23]. Determination of onset timing by phase detection, rather than via percentage of gait cycle assessment, allowed the synchronization of assistive torque with the wearer's motion regardless of climbing speed changes. To prevent assistive torque for level-ground walking during the stair climb, the assistance algorithm assessed the current ground state. The workflow of stair-climbing assistance is shown in Figure 3.

The *τ*_*p*_ and *t*_*p*_, not optimized for each subject, were set empirically using preliminary experiments (Table 1). The assistive torques defined in the time domain were equally applied to all subjects after initiation of motion. However, their application varied in a subject-specific manner based on stair-climbing speed and stance cycles (Figure 4).

### 2.4. Experimental Protocol

The subjects were asked to rest for at least 5 min in a sitting position. Subsequently, oxygen consumption and heart rates were measured for 2 min in a standing position using a portable metabolic system (K4b2, COSMED, Rome, Italy) and a heart rate monitor (TICKR X, Wahoo, Atlanta, United States), respectively. Following the establishment of the resting heart rate (±5 beats per min), the subjects climbed nine flights of stairs (total of 195 steps; 20 steps per level through the 7th floor and 25 steps per level from the 7th floor to the 10th floor) twice at a self-selected speed. One trial was carried out without assistance (i.e., zero-impedance mode), with stair-climbing assistance applied for the other trial, and the order of trials was randomized. Subjects rested for at least 10 min between trials. During climbing, oxygen consumption, heart rate, and time to climb each level were measured. A practice period was provided to help subjects adapt to the wearable robot, with a maximum of two practice periods allowed.

### 2.5. Data Processing

A custom *m*-file (MATLAB, MathWorks, Natick, MA, USA) was used for data processing. Oxygen consumption and heart rate values were smoothed to eliminate measurement noise and outliers using smooth.*m*, with span = 10%, and method = rloess, where span is the length of the moving window as a percentage of the raw data, with the rloess method applying a second-order regression to the raw data from which the outlier is excluded [31]. Net oxygen cost (NOC) was calculated as the difference between the oxygen consumption rate and the average resting oxygen consumption rate divided by the stair-climbing speed [32]. Total heart beats (THB) [33] during the climbing session were calculated by numerical integration of the heart rate. The average climbing speed was calculated by dividing the number of steps by the climbing time. NOC, THB, and average climbing speed of the two climbing trials were compared using a paired *t*-test, with *P* values < 0.05 considered statistically significant. The paired *t*-test was performed using SPSS ver. 24 (SPSS Inc., Chicago, IL, USA).

## 3. Results and Discussion

### 3.1. Results

On average, stair-climbing assistance reduced NOC and THB by 9.3% (*P* < 0.001) and 6.9% (*P* = 0.003), respectively (Figure 5). For all subjects, although the average speed per level varied during climbing, no significant between-trial differences were observed (Figure 6).

## 4. Discussion

### 4.1. Stair-Climbing Speed

In contrast to previous studies utilizing treadmills, the present experiments were conducted using nine flights of physical stairs. Despite the lack of a controlled experimental environment with strict regulation of climbing speed and motion analysis, these results more closely reflect real-life circumstances. With the ability to self-select climbing speed, the subjects demonstrated individual and within-climb differences in ascent speeds. However, the ZIC and assist conditions did not result in significant differences in the average stair-climbing speeds. These results indicated that, under the conditions tested, stair-climbing assistance has no effect on climbing speed.

### 4.2. NOC Reduction

Multiple studies of exoskeleton assistance [3–11], utilizing a treadmill environment to regulate walking speed, evaluated steady-state values of oxygen consumption and heart rate as indices of metabolic cost. Presently, we also considered the self-selected climbing speed for the assessment of metabolic cost. Plasschaert et al. previously defined NOC as the difference between the average oxygen consumption rate during walking and that during resting divided by the average walking speed [32]. Substituting the average climbing speed (steps/min) into the equation, we found that the metabolic cost decreased by 9.3% in the presence of stair-climbing assistance.

### 4.3. THB Reduction

In a manner similar to NOC, the heart rate should also be analyzed in a nonsteady state induced by climbing speed changes. Hood et al. defined the THB index as the ratio of THB during the exercise period to the total traveled distance [33]. As the subjects covered the same climbing distance in the present study, unadjusted THB values were considered. In addition to serving as an accurate and convenient estimate of energy expenditure, the heart rate also directly reflects the cardiac burden of a person. Presently, THB decreased by 6.9% following robotic exoskeleton assistance, suggesting that climbing assistance can reduce cardiovascular burden.

### 4.4. Methodological Issues and Limitations

The present study used a trunk-hip-knee-ankle-foot- (THKAF-) type multijoint robotic exoskeleton [34]. Exoskeletons of this type have been used to provide full assistance to paraplegic patients to move their legs. Using such exoskeletons on nondisabled wearers requires the exoskeletal joints to have zero impedance, or zero torque [35]. Ankle exoskeletons for walking assistance have provided energetic cost advantages due to negligible device weight and minimal interference in joint function. Multijoint soft exosuits, utilizing special actuation and power transmission mechanisms, have also considerably reduced metabolic costs due to limited weight and minimized resistive force. During stair climbing, the function of the knee joint (i.e., torque, power, and work) supersedes that of other joints [14], with most exoskeletons for stair-climbing assistance previously developed as knee-type devices. Thus, stair-climbing assistance using a THKAF-type exoskeleton was expected to be effective for metabolic cost reduction.

Despite its considerable weight, the THKAF-type exoskeleton was sufficiently portable to perform experiments using a physical stair environment. However, our experiments were limited in their ability to obtain data for biomechanical analyses, including measurements of muscle activity and of human motion in a three-dimensional space. Lack of kinematic and kinetic information, as well as of electromyography data, represents a limitation of this study that hinders direct comparisons with other works. Despite this drawback, this study demonstrated, for the first time, reduction in climbing-associated energy consumption using a THKAF-type exoskeleton.

Presently, equal assistive torque was provided to all subjects, with parameters (Table 1) empirically determined using preliminary studies. However, subject-specific assistive torque parameters may maximize the assistance effect for individual subjects. Recent studies have demonstrated that optimization of individual assistive force profiles can further reduce energy consumption [11, 36]. Thus, subject-specific optimization of the assistive torque provided by the exoskeleton tested here may result in improved climbing assistance effects. However, despite identical assistive torques, the present study demonstrated effective stair-climbing assistance for all subjects.

Multiple studies have compared metabolic costs between robotic assistance and no-robot or unpowered conditions [5, 8, 9, 36, 37]. However, the use of nondisabled subjects proficient in performing the tested physical tasks unassisted can mask the effects of assistance. The assistance effect can only emerge when the assistance overcomes the negative effects on energy consumption of factors such as exoskeleton weight, robot-imposed limitations in joint degree of freedom, and resistive forces of robotic joints [35]. Ding and colleagues [8, 36] used a tethered actuation system to facilitate assistance without increasing the weight load on the subjects. In cases where power sources could not be separated from the robot body, unpowered conditions have been used as controls to identify the assistance effect [5, 37]. However, it is also necessary to guarantee compliance of the robotic joints using specific mechanisms or control algorithms. Presently, as the actuation parts of the exoskeleton could not be separated from the robot body, ZIC was applied to ensure compliance of the robotic joints, with the metabolic cost compared to that under conditions of applied assistance. Thus, the possibility that the exoskeleton increases metabolic costs relative to no-robot conditions represents another limitation of this study. Such limitations, reported in other studies [3, 4], can be addressed by reducing exoskeleton weight, improving wearability, and ensuring greater degree of freedom of leg joints.

## 5. Conclusions

Stair-climbing assistance provided by an exoskeleton that assists flexion and extension of hip and knee joints reduced the metabolic cost and cardiovascular burden in healthy young males climbing nine floors of stairs.

## Figures and Tables

**Figure 1:** A robotic exoskeleton for lower limb assistance. DOF: degree of freedom; AFO: ankle-foot orthosis; F/E: flexion/extension.

**Figure 2:** Reduced mechanical impedance (resistive force) on the knee joint of the robotic exoskeleton after applying ZIC: (a) an arbitrary motion applied to the joint; (b) a resistive force against motion inputs; (c) a mechanical impedance defined as the magnitude of the ratio of the resistive force to the joint velocity in the frequency domain.

**Figure 3:** Workflow schematic of the stair-climbing assistance provided by the robotic exoskeleton. ZIC: zero-impedance control.

**Figure 4:** Example of knee extension torque for different stance times with the same *t*_*p*_ (0.25 s). AVG and STD indicate the mean and standard deviation of the stance time of the subject, respectively.

**Figure 5:** Stair-climbing net oxygen cost (NOC) and total heart beats (THB). NOC (a) and THB (b) were calculated for a 9-level stair climb with (ASSIST) and without climbing assistance (ZIC).

**Figure 6:** Average climbing speed. Climbing speed was measured under zero-impedance control (a) or climbing assistance (b) conditions.

**Table 1:** Defined assistive torque parameters. *τ*_*p*_: peak value of the assistive torque; *t*_*p*_: time taken to reach the *τ*_*p*_.

Joint	Stance phase		Swing phase	
	*τ*_*p*_	*t*_*p*_	*τ*_*p*_	*t*_*p*_
Hip	-27 Nm	0.25 s	16 Nm	0.2 s
Knee	-29 Nm	0.25 s	12 Nm	0.2 s

## Data Availability

The data used to support the findings of this study are available from the corresponding author upon request.
